# Positive Relationship between Serum Low-Density Lipoprotein Cholesterol Levels and Visceral Fat in a Chinese Nondiabetic Population

**DOI:** 10.1371/journal.pone.0112715

**Published:** 2014-11-14

**Authors:** Yuqi Luo, Xiaojing Ma, Yun Shen, Yaping Hao, Yaqin Hu, Yunfeng Xiao, Yuqian Bao, Weiping Jia

**Affiliations:** 1 Department of Endocrinology and Metabolism, Shanghai Jiao Tong University Affiliated Sixth People's Hospital; Shanghai Clinical Center for Diabetes; Shanghai Key Clinical Center for Metabolic Disease; Shanghai Diabetes Institute; Shanghai Key Laboratory of Diabetes Mellitus, Shanghai 200233, China; 2 Department of Radiology, Shanghai Jiao Tong University Affiliated Sixth People's Hospital, Shanghai 200233, China; University of Hong Kong, China

## Abstract

**Background:**

It has been reported that obesity and serum low-density lipoprotein cholesterol (LDL-c) are important risk factors of cardiovascular disease (CVD). It is recognized that regionalized adiposity has different cardiovascular risk, visceral versus subcutaneous, is a better predictor of CVD. However, the relationship between regionalized adiposity and LDL-c is unclear. The present study was designed to investigate the relationship between visceral fat accumulation and serum LDL-c levels in a Chinese cohort.

**Methods:**

A total of 1 538 subjects (539 men, 999 women; 20–75 years old) with normal glucose tolerance and blood pressure were recruited. All subjects underwent magnetic resonance imaging to quantify visceral fat area (VFA) and subcutaneous fat area. Serum LDL-c levels were detected by direct assay method.

**Results:**

Overweight/obese subjects (body mass index (BMI) ≥25 kg/m^2^) had significantly higher serum LDL-c levels than the lean subjects (BMI <25 kg/m^2^) (*P*<0.01). An increasing trend in serum LDL-c levels was found to accompany the increase in VFA (*P* for trend <0.01). Within the same BMI category, subjects with abdominal obesity (VFA ≥80 cm^2^) had significantly higher LDL-c levels than those without abdominal obesity (VFA <80 cm^2^) (*P*<0.05). Multiple stepwise regression analysis showed that increased VFA was an independent risk factor for elevated LDL-c levels, not only in the entire study population (*Standard β* = 0.138; *P*<0.01), but also when the study population was subdivided into men, premenopausal and postmenopausal women (*Standard β* = 0.117, 0.145, 0.090 respectively for men, premenopausal women, postmenopausal women; all *P*<0.01).

**Conclusions:**

VFA was positively correlated with serum LDL-c levels in a nondiabetic Chinese population with normal blood pressure.

## Introduction

Obesity is a worldwide epidemic and is closely associated with risk factors for cardiovascular disease (CVD), including hypertension, hyperglycemia, atherogenic dyslipidemia and metabolic syndrome (MetS). While total body fat contributes to whether or not a person is classified as obese, recent studies have shown that the pattern of fat distribution may be more predictive of the risk for atherosclerosis. Specifically, visceral fat accumulation has been shown to contribute to atherosclerosis pathogenesis [1], [2].

Previous research has shown that hypercholesterolemia, low high-density lipoprotein cholesterol (HDL-c) levels and elevated serum low-density lipoprotein cholesterol (LDL-c) levels are prerequisites for atherogenesis [2]. Moreover, people with elevated LDL-c levels are at higher risk for CVD [3], [4]. In guidelines established for the prevention and treatment of CVD, lipid-lowering therapies are recommended specifically to lower LDL-c levels and reduce risk for CVD [5], [6].

Although independent roles for visceral fat accumulation and elevated serum LDL-c in atherosclerosis have been recognized, it is unclear whether these factors are associated with one another. The relationship between visceral fat accumulation and LDL-c is poorly understood in part due to a paucity of large community-based studies on visceral fat area (VFA), specifically in a Chinese population. Moreover, previous studies that have addressed the relationship of visceral fat to LDL-c have predominantly been performed in cohorts with CVD [7], [8]. Because CVD patients may already be receiving anti-diabetic, antihypertensive or lipid-lowering therapies, lipid levels and lipoprotein metabolism may be altered and confound the analysis. To better address the relationship between visceral fat accumulation and serum LDL-c levels, this study was designed to analyze a Chinese population with normal glucose tolerance and normal blood pressure while excluding subjects currently receiving treatment for dyslipidemia.

## Subjects and Methods

### Ethics Statement

The whole study was conducted in accordance with the Declaration of Helsinki and approved by the Ethics Committee of Shanghai Jiao Tong University Affiliated Sixth People's Hospital. All study participants provided written informed consent prior to enrollment.

### Subjects

The subjects for this study were selected from the Shanghai Obesity Study (SHOS). The details for the SHOS study population have been previously published [9]. From December 2009 to December 2011, 1 908 subjects with normal glucose tolerance and normal blood pressure were recruited to the study and underwent magnetic resonance imaging (MRI). A questionnaire was distributed to participants to acquire patient history on present or previous illness, medications taken, socioeconomic and lifestyle factors. Subjects were excluded from this study for the following reasons: currently incomplete anthropometric or laboratory data; taking medication for hyperlipidemia; hepatic or renal dysfunction; presence of malignant tumors; hyper- or hypothyroidism; known CVD history; currently treated with systemic corticosteroids; presence of a mental disorder; severe disability; hematological abnormalities or anemia; currently battling infection or C-reactive protein (CRP) levels >10 mg/L. After applying the above exclusion criteria, 1 538 subjects between 20 and 75 years of age remained in this study.

### Anthropometric and Laboratory measurements

Body mass index (BMI) was determined as subject weight divided by height squared. Waist circumference (W) measurements were acquired at the horizontal plane between the inferior costal margin and the iliac crest on the mid-axillary line. Systolic blood pressure (SBP) and diastolic blood pressure (DBP) were calculated by taking the average of three measurements over a period of three-minute intervals using a mercury sphygmomanometer.

A same 3.0. T clinical MRI scanner (Archiva, Philips Medical System, The Netherlands) was used to acquire data on VFA and subcutaneous fat area (SFA). The MRI scanner was conducted by an experienced radiological technician blind to the results. MRI images were obtained at the abdominal level between lumbar 4 and lumbar 5 vertebrae in the supine position. Two trained observers unaware of the results used SLICE-O-MATIC image analysis software (version 4.2; Tomovision Inc., Montreal, QC, Canada) to split the images into VFA and SFA. A third observer who did not know the results would reanalyzed the image, once results of the same one differed by more than 10% [10].

All patients were subjected to a 75 g oral glucose tolerance test (OGTT). Blood samples were collected after a 10 h overnight fast to measure fasting plasma glucose (FPG) and 2 h post-OGTT plasma glucose (2hPG) by using a standard glucose oxidase method. Glycated hemoglobin (HbA1c) level was determined by high-pressure liquid chromatography (Bio-Rad Inc., Hercules, CA, USA). A radioimmunoassay (Roche Diagnostics GmbH, Mannheim, Germany) was used to measure fasting serum insulin (FINS), with intra- and inter-assay coefficients of variation of 1.7% and 2.5%, respectively. The Homeostasis Model of Assessment-Insulin Resistance (HOMA-IR) was then calculated to estimate insulin sensitivity as follows: (FPG [mmol/L] × FINS [mU/L])/22.5 [9]. Serum lipid profiles, including total cholesterol (TC), triglycerides (TG), HDL-c, LDL-c, apolipoprotein B (ApoB) and lipoprotein a (Lp(a)) were measured with a 7600-120 Hitachi automatic analyzer (Hitachi, Tokyo, Japan). TC and TG were measured enzymatically (Roche Diagnostics GmbH) while HDL-c and LDL-c were measured using a direct assay method (Sekisui Medical Co., Ltd., Tokyo, Japan). ApoB was detected using an immunoturbidimetric approach (Kehua Bio-engineering Co., Ltd., Shanghai, China) and latex agglutination turbidimetry (Sekisui Medical Co., Ltd.) was used to measure Lp(a) levels. CRP was detected using a scattering turbidimetric approach (Siemens Healthcare Diagnostic Inc., Newark, NJ, USA).

### Diagnostic Definition

Normal glucose tolerance was defined according to the criteria established by the 1999 World Health Organization (WHO), which FPG was less than 6.1 mmol/L and 2hPG was less than 7.8 mmol/L [11]. Normal blood pressure was defined according to the 1999 WHO/International Society of Hypertension (ISH) hypertension guidelines, with a SBP less than 130 mmHg and a DBP less than 85 mmHg [12]. The 1998 WHO standards were used to classify BMI, a subject with a BMI ≥25 kg/m^2^ was classified as overweight/obese while subjects with BMI <25 kg/m^2^ were classified as lean [13]. Based on the results from our previous study, subjects with a VFA ≥80 cm^2^ were classified as visceral obesity [14]. The Third Report of the Expert Panel on Detection, Evaluation, and Treatment of High Blood Cholesterol in Adults was used to diagnose dyslipidemia as follows: serum TC levels ≥6.22 mmol/L, and/or serum TG levels ≥2.26 mmol/L, and/or serum HDL-c levels <1.04 mmol/L, and/or serum LDL-c levels ≥4.14 mmol/L [5]. Current cigarette smokers were defined as subjects who smoked at least one cigarette per day for longer than six months [9].

### Statistical Analysis

All statistical analyses were performed using the SPSS statistical software, version 16.0 (SPSS, Chicago, IL, USA). Subject data with normal distribution were presented as the mean ± standard deviation (SD) while data lacking normal distribution were presented as the median (inter-quartile range 25–75%). To analyze trends, a one-way analysis of variance (ANOVA) was used. Intergroup comparisons of normally distributed clinical data were assessed with an unpaired student's *t* test, while the Mann-Whitney U test was applied for data lacking normal distribution. A chi-square test was used for intergroup comparisons between categorical variables. Spearman and partial correlation analysis were used to assess the relationship between VFA and the clinical variables. A multivariate regression analysis was carried out using a stepwise multiple regression model to evaluate the correlation between VFA and atherogenic lipoprotein cholesterol. All *P*-values were two-tailed and a *P*-value less than 0.05 was set as the threshold for statistical significance.

## Results

### Clinical characteristics of the study subjects

A total of 1 538 subjects (539 men, 999 women) from 20 to 75 years of age were included in the study. Of the 1 538 subjects, 379 subjects (24.6%) were diagnosed with dyslipidemia, wherein 177 (11.5%) had elevated serum LDL-c levels. The clinical characteristics of the study subjects are shown in Table 1. When compared to the lean subjects (BMI <25 kg/m^2^), the overweight/obese subjects (BMI ≥25 kg/m^2^) had a significantly higher serum LDL-c and ApoB levels. Moreover, the overweight/obese subjects also had significantly higher W, VFA, SFA, SBP, DPB, blood glucose, HOMA-IR, TG and CRP (all *P*<0.05).

**Table 1:** Clinical characteristics of the subjects subdivided by BMI.

Variables	Total	BMI <25 kg/m^2^	BMI ≥25 kg/m^2^	*P*
n	1538	1245	293	-
Age (years)	51.7(44.9–56.9)	51.9(45.0–56.9)	50.0(44.6–56.9)	0.32
BMI (kg/m^2^)	22.7±2.8	21.7±2.0	26.9±1.6	<0.01
W (cm)	78.0(72.0–84.0)	76.0(71.0–81.0)	88.5(83.8–93.5)	<0.01
VFA (cm^2^)	62.8(44.5–87.7)	56.7(40.9–76.8)	95.9(75.0–127.7)	<0.01
SFA (cm^2^)	161.2(121.6–202.9)	150.2(114.2–186.9)	211.7(170.0–257.6)	<0.01
SBP (mmHg)	116.0(108.0–120.7)	114.7(107.3–120.7)	120.0(110.0–122.0)	<0.01
DBP (mmHg)	73.3(69.3–79.3)	72.7(69.3–79.3)	76.7(70.0–79.7)	<0.01
FPG (mmol/L)	5.1±0.4	5.1±0.4	5.2±0.4	<0.01
2hPG (mmol/L)	5.8±1.1	5.8±1.0	5.9±1.1	0.04
HbA1c (%)	5.5(5.3–5.7)	5.5(5.3–5.7)	5.6(5.3–5.8)	<0.01
FINS (mU/L)	6.7(4.9–9.4)	6.3(4.5–8.5)	9.6(6.7–13.1)	<0.01
HOMA-IR	1.5(1.1–2.2)	1.4(1.0–2.0)	2.2(1.5–3.1)	<0.01
TC (mmol/L)	4.96(4.36–5.62)	4.95(4.36–5.66)	4.97(4.36–5.55)	0.44
TG (mmol/L)	1.10(0.78–1.55)	1.04(0.75–1.48)	1.35(0.99–1.84)	<0.01
HDL-c (mmol/L)	1.47(1.25–1.75)	1.51(1.28–1.77)	1.33(1.13–1.54)	<0.01
LDL-c (mmol/L)	3.11(2.57–3.66)	3.06(2.54–3.65)	3.27(2.73–3.72)	<0.01
ApoB (g/L)	0.78(0.68–0.89)	0.78(0.67–0.89)	0.80(0.70–0.91)	<0.01
Lp(a) (mg/dL)	10.60(6.30–20.35)	10.80(6.40–20.40)	9.94(5.65–18.35)	0.15
CRP (mg/L)	0.5(0.3–1.1)	0.5(0.2–0.9)	0.8(0.4–1.6)	<0.01
Dyslipidemia, N (%)	379(24.6)	302(24.3)	77(26.3)	0.47
hypercholesterolemia, N (%)	158(10.3)	142(11.4)	16(5.5)	<0.01
hypertriglyceridemia, N (%)	129(8.4)	93(7.5)	36(12.3)	<0.01
Low HDL-c, N (%)	98(6.4)	70(5.6)	28(9.6)	0.01
High LDL-c, N (%)	177(11.5)	150(12.0)	27(9.2)	0.17
Diabetes family history, N (%)	311(20.2)	246(19.8)	65(22.2)	0.35
CVD family history, N (%)	426(27.7)	349(28.0)	77(26.3)	0.55
Dyslipidemia family history, N (%)	225(14.6)	179(14.4)	46(15.7)	0.56
Current smoker, N (%)	347(22.6)	259(20.8)	88(30.0)	<0.01

ApoB: apolipoprotein B; 2hPG: 2-h post-OGTT plasma glucose; BMI: body mass index; CRP: C reactive protein; CVD: cardiovascular disease; DBP: diastolic blood pressure; FINS: fasting insulin; FPG: fasting plasma glucose; HbA1c: glycated hemoglobin; HDL-c: high-density lipoprotein cholesterol; HOMA-IR: homeostasis model assessment-insulin resistance; LDL-c: low-density lipoprotein cholesterol; Lp(a): lipoprotein a; SBP: systolic blood pressure; SFA: subcutaneous fat area; TC: total cholesterol; TG: triglyceride; VFA: visceral fat area; W: waist circumference.

Data are presented as means ± SD or median (interquartile range 25–75%) or N (%). *P* for BMI ≥25 kg/m^2^ versus BMI <25 kg/m^2^.

In the overweight/obese group, we observed a significant increase in the frequency of dyslipidemia, which included hypercholesterolemia, hypertriglyceridemia and low HDL-c (all *P*<0.05). The frequency of high LDL-c between the lean and overweight/obese groups, however, did not show statistical significance (*P*>0.05). It is important to note that there were more subjects who currently smoked in the overweight/obese group.

### Relationship between VFA and serum lipid profiles

Study subjects were divided into six VFA groups in 20 cm^2^ intervals, ranging from <40 cm^2^ to ≥120 cm^2^. Serum LDL-c and ApoB levels increased with an increase in VFA (LDL-c median for each group: 2.79, 2.96, 3.20, 3.15, 3.33, 3.42 mmol/L respectively, *P*-value for trend <0.01; ApoB median for each group: 0.71, 0.77, 0.81, 0.80, 0.83, 0.85 g/L respectively, *P* value for trend <0.01) (Figure 1). We observed an increasing trend for serum TC and TG levels with an increase in VFA (all *P*<0.01). A decreasing trend for serum HDL-c levels accompanied an increase in VFA (all *P*<0.01).

**Figure 1:** Distribution of serum LDL-c and ApoB levels with different VFA categories. Subjects were divided into six VFA subgroups from VFA <40 cm^2^ to VFA ≥120 cm^2^, according to 20 cm^2^ increments of VFA. *P*<0.01 for trend of elevated serum LDL-c and ApoB levels with increasing level of VFA. The bars represent median, 25th, and 75th percentile of LDL-c and ApoB levels.

To further evaluate how VFA levels were related to serum lipid and lipoprotein profiles, the lean and overweight/obese groups were subdivided based on the VFA cut-off point (VFA ≥80 cm^2^). In the lean group (BMI <25 kg/m^2^), subjects with a VFA ≥80 cm^2^ had significantly higher serum TC (5.09 [4.55–5.78] versus 4.92 [4.34–5.60] mmol/L; *P*<0.01), TG (1.46 [1.04–2.01] versus 0.96 [0.70–1.32] mmol/L; *P*<0.01), LDL-c (3.28 [2.77–3.75] versus 3.01 [2.49–3.59] mmol/L; *P*<0.01) (Figure 2A), ApoB (0.82 [0.72–0.92] versus 0.77 [0.66–0.88] g/L; *P*<0.01) (Figure 2 B) and lower serum HDL-c levels (1.31 [1.14–1.50] versus 1.57 [1.34–1.82] mmol/L; *P*<0.01) than the subjects with a BMI <25 kg/m^2^ and a VFA <80 cm^2^. We observed a similar trend in the overweight/obese group (BMI ≥25 kg/m^2^) subdivided for VFA. Overweight/obese subjects with a VFA ≥80 cm^2^ had significantly higher serum TC (5.03 [4.48–5.57] versus 4.70 [4.15–5.44] mmol/L; *P*<0.05), TG (1.48 [1.09–2.00] versus 1.11 [0.78–1.40] mmol/L; *P*<0.01), LDL-c (3.30 [2.84–3.76] versus 3.09 [2.57–3.66] mmol/L; *P*<0.05) (Figure 2 A), ApoB (0.82 [0.73–0.92] versus 0.76 [0.67–0.86] g/L; *P*<0.01) (Figure 2 B), and lower serum HDL-c levels (1.27 [1.10–1.49] versus 1.45 [1.21–1.70] mmol/L; *P*<0.01) than the overweight/obese subjects with a VFA <80 cm^2^. However, Lp(a) levels of subjects did not reach statistical significance between the VFA <80 cm^2^ subgroup and VFA ≥80 cm^2^ subgroup (*P*>0.05), not only in the BMI <25 kg/m^2^ group but also in the BMI ≥25 kg/m^2^ group.

**Figure 2:** Serum LDL-c and ApoB levels with different VFA levels in the same BMI categories. A: Within the same BMI category, serum LDL-c levels of subjects with VFA ≥80 cm^2^ were significantly higher than those with VFA <80 cm^2^ (*P*<0.01 in BMI <25 kg/m^2^; *P*<0.05 in BMI ≥25 kg/m^2^). B: Within the same BMI category, serum ApoB levels of subjects with increased visceral fat (VFA ≥80 cm^2^) were significantly higher than those with VFA <80 cm^2^ (all *P*<0.01).

### Factors affecting serum LDL-c levels

To evaluate the association between VFA and the clinical parameters, a Spearman correlation analysis was performed. VFA was positively correlated with LDL-c levels (*P*<0.01). To determine whether total body fat affected the correlation between VFA and LDL-c, a partial correlation analysis was conducted after making adjustments for age, gender and BMI (Table 2). Even after adjustments, VFA was still positively correlated with LDL-c (*P*<0.01). In addition, VFA was also positively correlated with W, FPG, 2hPG, FINS, HOMA-IR, TC, TG, ApoB and CRP (all *P*<0.05), but negatively correlated with HDL-c (*P*<0.01).

**Table 2:** Spearman and partial correlation analysis of VFA.

Variables	VFA		VFA (Adjusted of age, gender and BMI)^a^	
	r	*P*	r	*P*
BMI	0.665	<0.001	-	-
W	0.724	<0.001	0.396	<0.001
SBP	0.139	<0.001	−0.010	0.691
DBP	0.108	<0.001	0.026	0.318
FPG	0.167	<0.001	0.066	<0.05
2hPG	0.175	<0.001	0.121	<0.001
HbA1c	0.120	<0.001	0.027	0.284
FINS	0.334	<0.001	0.164	<0.001
HOMA-IR	0.341	<0.001	0.166	<0.001
TC	0.150	<0.001	0.151	<0.001
TG	0.468	<0.001	0.292	<0.001
HDL-c	−0.400	<0.001	−0.178	<0.001
LDL-c	0.237	<0.001	0.135	<0.001
ApoB	0.259	<0.001	0.171	<0.001
Lp(a)	−0.043	0.091	−0.008	0.756
CRP	0.411	<0.001	0.144	<0.001

ApoB: apolipoprotein B; 2hPG: 2-h post-OGTT plasma glucose; BMI: body mass index; CRP: C reactive protein; DBP: diastolic blood pressure; FINS: fasting insulin; FPG: fasting plasma glucose; HbA1c: glycated hemoglobin; HDL-c: high-density lipoprotein cholesterol; HOMA-IR: homeostasis model assessment-insulin resistance; LDL-c: low-density lipoprotein cholesterol; Lp(a): lipoprotein a; SBP: systolic blood pressure; TC: total cholesterol; TG: triglyceride; W: waist circumference.

a Partial correlation: adjusted of age, gender and BMI.

To further investigate the independent association between VFA and LDL-c, a multiple stepwise regression analysis was performed (Table 3). Because lipid profile levels are greatly influenced by factors such as gender and menopausal status, we subdivided the total study population into men, premenopausal women and postmenopausal women. LDL-c was set as the dependent variable, while age, BMI, W, VFA, SFA, SBP, DBP, FPG, 2hPG, FINS, TG, HDL-c, CRP, smoking status, CVD family history and dyslipidemia family history were designated as the independent variables to be assessed in all groups. We found that VFA was independently associated with LDL-c, both in the entire study population (Standard β = 0.138; *P*<0.01) and after subdivision of the subjects (Standard β = 0.138, 0.136 and 0.129 for men, premenopausal women and postmenopausal women, respectively; all *P*<0.01). In addition, the age, FINS and smoking status in men, the age, FINS and HDL-c levels in premenopausal women, the TG and HDL-c levels in postmenopausal women were identified as independent risk factors for LDL-c (all *P*<0.01).

**Table 3:** Multiple stepwise regression analyses of serum LDL-c.

Independent variables	β coefficient	Standard error	Standard β	*P*
Total				
Age	0.021	0.002	0.225	<0.001
VFA	0.003	0.001	0.138	<0.001
FINS	0.034	0.006	0.157	<0.001
TG	0.069	0.031	0.065	0.024
HDL-c	0.337	0.065	0.148	<0.001
Smoking status	0.058	0.025	0.060	0.019
Men				
Age	0.014	0.004	0.153	<0.001
VFA	0.003	0.001	0.138	0.003
FINS	0.039	0.010	0.178	<0.001
Smoking status	0.106	0.039	0.112	0.007
Premenopausal Women				
Age	0.026	0.005	0.230	<0.001
VFA	0.004	0.002	0.136	0.005
HDL-c	0.288	0.107	0.123	0.008
FINS	0.037	0.008	0.204	<0.001
Postmenopausal Women				
VFA	0.004	0.001	0.129	0.006
TG	0.146	0.056	0.137	0.009
HDL-c	0.418	0.107	0.197	<0.001

FINS: fasting insulin; HDL-c: high-density lipoprotein cholesterol; TG: triglyceride; VFA: visceral fat area.

Independent variables: Age, BMI, W, VFA, SFA, SBP, DBP, FPG, 2hPG, FINS, TG, HDL-c, CRP, smoking status, CVD family history, dyslipidemia family history.

## Discussion

In recent years, and especially in developing nations, CVD has become the leading cause of death. A primary contributor to CVD is atherosclerosis, with plaque formation caused by accumulation of lipoprotein deposits in the arterial walls. One of the predominant risk factors for atherogenesis is elevated LDL-c levels [15] and ApoB, the primary apolipoprotein component accounting for approximately 97% of the total LDL protein particles, and its levels may be indicative of the potential atherogenic lipoprotein particles [16], [17].

Results from the Framingham Heart Study demonstrated that obesity is a critical risk factor for CVD [18]. It has been reported that abdominal or visceral obesity may have a higher atherogenic potential than general obesity [19]. Recent studies have demonstrated that increased visceral adipose is closely associated with these atherogenic factors across different study populations. For example, Demerath et al. [20] found that, after adjusting for age, serum LDL-c levels increased with increasing VFA in non-Hispanic whites.

A previous cross-sectional study found that among anthropometrics and imaging indices of obesity, waist circumference showed a stronger association with dyslipidemia in patients with CVD, while computed tomography (CT)-measured VFA was more strongly associated with dyslipidemia in patients without CVD [8]. Thus, compared to waist circumference, VFA was a better prognostic indictor for early signs of abnormal metabolic profiles. A small domestic study of 108 cardiovascular inpatients found a positive correlation between CT-measured VFA and LDL-c, however its small sample size and high risk subjects limit the ability to generalize the study's findings. A significantly larger study with 47 325 participants performed by the China National Diabetes and Metabolic Disorders Study found that serum LDL-c levels elevated with the increment of BMI and waist circumference [21]. Although waist circumference is a convenient factor for measurement, it does not distinguish subcutaneous adiposity from visceral adiposity and does not allow an evaluation of how abdominal fat accumulation specifically relates to atherogenesis and CVD.

Because of the limitations of the above studies in addressing the specific role of visceral fat in atherogenesis, we designed a large, community-based study with a population lacking the confounding factors of glycometabolism disorders. What's more, we implemented MRI to accurately measure visceral fat deposition. Both CT and MRI are recommended by international diabetes federation as the platinum standards to evaluate adipose deposition [22]. With the capacity to distinguish adipose tissue from other tissue by density, CT scanning has been frequently used for measuring visceral fat. However, it results in exposure to ionizing radiation. MRI scanning gains its advantage in identifying soft tissue owing to superior fat-water separation quality. Moreover, without radiation exposure, MRI has been more widely used to measure visceral fat content recently. Although the imaging properties of CT and MRI differed, Klopfenstein et al. [23] found good agreement between the two methods when measuring VFA in 27 polycystic ovarian syndrome women. Therefore, MRI is a favourable, non-radiation-exposing alternative for measuring VFA in clinical practice and research. From our analysis, we found that elevated LDL-c and ApoB levels were associated with increases in BMI and increased MRI-measured VFA. The association between subjects with VFA ≥80 cm^2^ and higher levels of atherogenic lipoprotein cholesterol levels occurred independently of total body fat. It is important to note that, even with the same BMI, East Asians are more prone to visceral fat accumulation than Caucasians, indicating that racial diversities exist in body fat distribution [14].

Gender-related differences might also exist in body fat distribution and lipid metabolism. In a study of Canadian men, Lemieux et al. [24] found that CT-measured VFA was positively correlated with serum LDL-c levels. A one-year lifestyle intervention study of 107 non-diabetic, abdominally obese Caucasian men found that a reduction of ApoB was accompanied by a significant decrease in VFA [25]. A study of 157 subjects with a high prevalence (34%) of MetS from Onat and colleagues [26] found that ApoB levels were independently associated with VFA in men, but not in women. Thus, our study was designed to further evaluate whether increased VFA was independently associated with increased LDL-c across gender subgroups. Our analysis identified VFA as an independent risk factor for elevated serum LDL-c across the entire study population, after adjusting for confounding factors, and in distinct gender subgroups.

There are several reasons for the positive association between elevated VFA and LDL-c. Bjorntorp et al. [27] demonstrated that an increase in visceral adipose tissue can lead to extensive lipolysis, a process that is mediated through insulin resistance. Excess FFA are exported from abdominal adipose tissue are thought to be a triggering factor for TG synthesis in the liver. Prolonged exposure to elevated FFA leads to increased HDL-c synthesis and concomitantly, an increase in LDL-c, an intermediate product of lipid metabolism and ApoB, which ultimately get released into the arterial system and deposited to trigger atherogenesis.

Lp(a) has LDL-like properties and it has been hypothesized that elevated Lp(a) could increase the risk for atherosclerosis. In support of this idea, studies have found that individuals with high Lp(a) levels are more likely to develop CVD [28], [29]. Recent studies, however, have found that serum Lp(a) levels are primarily determined by genetics, and rarely influenced by age, sex, or body weight [6]. In line with this finding, the present study did not identify a relationship between Lp(a) and VFA. A potential role for obesity in Lp(a)-associated pathogenesis remains to be elucidated.

There were two limitations to the present study. First, the cross-sectional nature of the study design precluded the capacity to evaluate a causal relationship between serum LDL-c levels and central obesity. Second, the study was conducted in a Chinese population with normal glucose tolerance and normal blood pressure, limiting the degree to which the findings can be generalized.

## Conclusions

Localized adipose accumulation in the abdomen and atherogenic factors are closely associated. An increase in VFA was positively correlated with increases in cardiovascular risk factors such as LDL-c.
